# Gastrodin protects retinal ganglion cells from ischemic injury by activating phosphatidylinositol 3-kinase/protein kinase B/nuclear factor erythroid 2-related factor 2 (PI3K/AKT/Nrf2) signaling pathway

This article has been retracted.

**DOI:** 10.1080/21655979.2022.2076499

**Published:** 2022-05-24

**Authors:** Sizhen Li, Qingsong Yang, Zixiu Zhou, Xiaodong Yang, Yating Liu, Kuanxiao Hao, Min Fu

**Affiliations:** Nanjing Tongren Eye Center, Nanjing Tongren Hospital, School of Medicine, Southeast University, Nanjing, P.R. China

**Keywords:** Gastrodin, apoptosis, oxidative stress, ischemic injury, PI3K/AKT/Nrf2 pathway

## Abstract

Glaucoma is a progressive optic neuropathy and improper treatment may cause irreversible damage to visual function. Gastrodin is an effective active substance extracted from Gastrodia elata and possesses antioxidant as well as anti-inflammatory properties. However, the therapeutic potential of gastrodin for retinal ischemia/reperfusion (I/R) injury remains unclear. We adopted oxygen and glucose deprivation/reoxygenation (OGD/R) to induce R28 cells with the aim of simulating glaucomatous neurodegeneration. CCK-8 analysis and TUNEL were applied for examining cell proliferation and apoptosis . In addition, RT-qPCR and ELISA were performed to test the releases of inflammatory factors in cells . Related indicators of intracellular oxidative stress and ROS production were detected by corresponding kits. Moreover, western blot was applied to assay the expressions of PI3K/AKT/Nrf2 pathway-related proteins. OGD/R induction contributed to the decreased cell viability and reduced Bcl-2 protein expression, while the protein contents of Bax, Cyto-C, c-caspase 9 and c-PARP as well as ROS production were ascended. The co-treatment of hypoxia and gastrodin greatly improved R28 cell viability but effectively suppressed cell apoptosis, ROS level and the releases of OGD/R-induced inflammatory factors as well as oxidative stress. In addition, OGD/R stimulation reduced Nrf2, accompanied by a decrease in the phosphorylation levels of PI3K and AKT. Gastrodin significantly promoted the activation of PI3K/AKT/Nrf2 signaling pathway in R28 cells, which was then counteracted by PI3K/AKT inhibitors. In conclusion, the present study suggested that gastrodin has a protective effect on OGD/R-induced R28 cell injury, which is achieved through the activation of the PI3K/AKT/Nrf2 signaling pathway.

## Highlights

- Gastrodin can ameliorate OGD/R-induced apoptosis, inflammatory response, and oxidative stress of R28 cells.
- Gastrodin can activate PI3K/AKT/Nrf2 signaling pathway
- PI3K/Akt inhibitor LY294002 can aggravate OGD/R-induced R28 cell injury

## Introduction

Glaucoma is a chronic progressive neurodegenerative disease characterized by persistent damage to retinal ganglion cells (RGCs), irreparable visual field defects and pathologically elevated intraocular pressure (IOP) [1,2]. The visual function damage caused by glaucoma is one of the main causes of blindness worldwide [3]. It is well known that retinal blood supply disorder, reperfusion injury, and nutritional deficiency caused by elevated IOP are considered to be the most important risk factors for the occurrence and development of glaucoma [4]. However, progressive optic nerve injury still occurs in some patients after drug intervention, laser therapy, or surgical treatment, which are only aimed to reduce IOP [5]. Therefore, in this case, it is urgent to find effective drugs that protect vision by preventing the death of retinal ganglion cells.

Gastrodin is an active ingredient extracted from traditional Chinese herbal medicine Gastrodia elata [6]. Researches have noted that gastrodin exhibits a variety of pharmacological properties, including anti-inflammation, anti-oxidative stress, and anti-apoptosis [7,8]. For example, gastrodin can regulate NLRP3/caspase-1 pathway by inhibiting the activity of NLRP3 inflammasomes and improving cell apoptosis caused by myocardial microvascular reperfusion injury [9]. Gastrodin treatment also reduced ROS production of macrophages and protected macrophages from oxidative stress-induced apoptosis [10]. Li et al. reported that gastrodin pre-treatment could significantly compensate for the ischemia-reperfusion (I/R)-induced inflammatory response and apoptosis, thereby reducing the damage caused by cerebral I/R in rats [11]. Zhang et al. demonstrated that gastrodin could inhibit high glucose-induced oxidative stress and apoptosis in human retinal endothelial cells by regulating SIRT1/TLR4/NF-κBp65 signaling pathway [12]. Notably, gastrodin has potential application value in the treatment of retinal neurodegenerative diseases characterized by retinal ganglion cell death [13]. However, no study has been conducted to investigate the biological function of gastrodin in retinal I/R injury.

PI3K/Akt/Nrf2 signaling pathway is a major player in a variety of biological processes by inhibiting pro-apoptotic signals and inflammation [14,15], while its role in I/R injury has been revealed in recent studies. Evidence from Wu et al. demonstrated that dexmedetomidine inhibited NLRP3 inflammatory corpuscles and alleviated liver I/R damage by activating PI3K/AKT/Nrf2 pathway [16]. Ginsenoside Rb1 alleviated I/R-induced intestinal inflammation and oxidative stress by activating PI3K/Akt/Nrf2 pathway [17], and edaravone protected retina from oxidative damage induced by I/R through PI3K/Akt/Nrf2 pathway [18]. Fortunately, increasing reports have shown that gastrodin can activate PI3K/AKT-related pathways to alleviate the hypoxic damage of cells. Li and his colleagues showed that gastrodin inhibited autophagy by activating mTOR signal in PI3K-Akt pathway and protected neonatal rat cardiomyocytes from hypoxia/reoxygenation injury [19]. Xing et al. reported that gastrodin activated PTEN/PI3K/AKT and NF-κB pathway by up-regulating miR-21, and alleviated the hypoxia injury of H9c2 cells [20]. Yuan et al. proved that gastrodin preconditioning could protect the liver from I/R injury by activating Nrf2/HO-1 pathway [21].

Collectively, we speculated that gastrodin may also play a protective role in retinal ganglion cell hypoxia/reoxygenation injury by activating PI3K/AKT/Nrf2, so as to find new therapeutic drugs for glaucoma.

## Materials and methods

***Cell culture*** Rat immortalized retinal precursor cells (R28) that were supplied by Beijing Crisprbio Biotechnology Co., LTD (Cat. No. CE19686) were grown in low-glucose DMEM medium (Gibco, USA, Cat. No 31,600,034), in which 10% Fetal Bovine Serum (Gibco; USA, Cat. No. 10,091,141) and 1% penicillin/streptomycin (Beyotiome, China, Cat. No C0222) were added. The incubator was supplied with 37°C and 5% CO_2_.

### Oxygen and glucose deprivation/reoxygenation (OGD/R) model and treatment

The OGD/R cell model was established according to a previous study [11]. Briefly, R28 cells were grown in low-glucose DMEM (Gibco, USA, Cat. No 31,600,034) and then transferred to a sealed hypoxic box containing 94% N_2_, 1% O_2_ and 5% CO_2_ and left for 4 h at 37°C. For re-oxygenation, the cells were cultured in normal MEM with 10% FBS and maintained for 24 h in reoxygenation under normoxic conditions. R28 cells which were cultured in complete medium (DMEM, 10% FBS) under normoxic conditions served as a control. After the incubation for 4 h under the condition of oxygen-glucose deprivation, Gastrodin (10, 25, 50, 100 μM) or 10 μM LY294002 (Sigma-Aldrich, Cas. No 934,389–88-5) were utilized to treat R28 cells in an incubator with 5% CO_2_ for 24 h. Cells that only treated with PBS served as a control.

#### Cell counting kit-8 (CCK-8) assay

R28 cells with a density of 5 × 10^3^ cells/well were inoculated in a 96-well cell culture plate and cultivated overnight at 37°C and 5% CO_2_. After the treatment with drugs for 24 h, 10 µl CCK-8 solution (Vazyme, Cat. No A311-01/02) was added to each well and the cells were cultivated for another 4 h at 37°C in 5% CO_2_. Cell viability evaluation was conducted by measuring absorbance at 450 nm with the use of a Varioskan™ LUX Multi-function microplate reader (Thermo Fisher Scientific, Inc.) [22].

#### Detection kit

All test kits used here were provided by Beyotime Biotechnology Co., Ltd. Lactate dehydrogenase cytotoxicity Test Kit (Cat. No. C0017) was used to detect the release of LDH in R28 cells to determine cytotoxicity in line with the guidelines of supplier. Lipid Oxidation (malondialdehyde, MDA) Detection Kit was performed to quantitatively detect the MDA level of R28 cells (Cat. No. S0131S) strictly as per reagent directions. After OGD/R stimulation, the levels of ROS and SOD in R28 cells with or without gastrodin treatment were detected by ROS detection kit (Cat. No. S0033S) and SOD activity detection kit (Cat. No. S0101M), respectively. Intracellular glutathione peroxidase activity was detected by corresponding assay kit (Cat. No. S0056). Enzyme-linked immunosorbent assay (ELISA) kit was employed to examine the levels of intracellular inflammatory factors TNF-α (Cat. No. PT516), IL-6 (Cat. No. PI328) and IL-1β (Cat. No. PI303).

#### TUNEL assay

The effects of gastrodin on the apoptosis of OGD/R-induced R28 cells were detected by TUNEL staining. In brief, cells (1x10^5^ cells/well) were rinsed by PBS for three times, followed by the fixation with 4% paraformaldehyde at room temperature. Subsequently, cells were probed with a small amount of DAPI staining (Beyotime, Cat. No. C1005) solution (covering the cells) and cultivated for 3–5 min at room temperature. 0.3% Triton-X-100 was also put into wells for further cultivation of cells. Afterward, 50 μl TUNEL assay solution (Beyotime, Cat. No. C1086) was employed to incubate the cells at 37°C in the dark for 60 min. Three fields of view were selected at random, and then cells were sealed with anti-fluorescence quenched sealing solution for observation under a fluorescence microscope (Zeiss GmbH, x200) [23].

#### Western blot

The R28 cells were cleaved with RIPA lysis buffer (Beyotime, Cat. No. P0013C) for 30 min on ice. Cell lysates were then collected and subjected to centrifugation (400 × g) at 4°C for 20 min. Protein supernatants in different groups were transferred to Eppendorf tubes. Determination of protein concentration was carried out using the Compat-Able™ BCA protein assay kit (Thermo Fisher Scientific, Inc; Cat. No. 23,229). Protein (40 µg) was subjected to 10% SDS-PAGE, transferred to PVDF membrane (Beyotime, Cat. No. FFP24) and sealed with 5% defatted milk powder at room temperature for 4 h. After washing for 3 times with 1x Tris Buffered Saline Tween, the membranes were incubated with following primary antibodies (all purchased from Abcam) against Bcl-2 (1:1,000; Cat. No. Ab194583), Bax (1:1,000; Cat. No. Ab32503), Cyto-C (1:1,000; Cat. No. Ab133504), Cleaved-caspase 9 (1:1,000; Cat. No. Ab2324), Cleaved-PARP (1:1,000; Cat. No. Ab32064), caspase 9 (1:1,000; Cat. No. Ab184768), PARP (1:1,000; Cat. No. ab227244), p-PI3K (1:1,000; Cat. No. Ab154598), p-AKT (1:1,000; Cat. No. Ab38449) and PI3K (1:1,000; Cat. No. Ab191606), Akt (1:1,000; Cat. No. Ab8805), Nrf2 (1:1,000; Cat. No. Ab92946) and GAPDH (1:1,000; Cat. No. ab181602) overnight at 4°C. Subsequently, the membranes were cultivated with goat anti-rabbit horseradish peroxidase conjugated IgG secondary antibody (1:1,000; Cat. No. Ab288151) for another 4 h at room temperature. Visualization of protein blots was undertaken with the application of enhanced chemiluminescence reagent (Thermo Fisher Scientific, Inc). Protein expression levels were semi-quantified using ImageJ software (version 1.8.0, National Institutes of Health) with GAPDH serving as the loading control [24].

#### Reverse transcription-quantitative PCR (RT-qPCR)

Extraction of total RNA from R28 cells was performed by RNAzol RT (Sigma-Aldrich; Merck KGaA), followed by the reverse transcription of RNA into cDNA with the help of a cDNA reverse transcription kit (Qiagen GmbH). Real-time PCR amplification was performed with the employment of SYBR Select Master Mix (Takara, Tokyo, Japan) on ABI7500 sequence detection system conforming to the manufacturer’s agreement. The primer sequences were listed as follows: TNF-α forward, 5′-ATGGGCTCCCTCTCATCAGT-3′, reverse, 5′-GCTTGGTGGTTTGCTACGAC-3′; IL-6 forward, 5′-CCAGTTGCCTTCTTGGGACT-3′, reverse, 5′-TGCCATTGCACAACTCTTTTC-3′; IL-1β forward, 5′-TCATCTTTGAAGAAGAGCCCG-3′, reverse, 5′-TCAGACAGCACGAGGCATTT-3′; GAPDH forward, 5′-TCCAACCCAACCCTCAACAG-3′, reverse, 5′-CCGATACGGCCAAATCCGTT-3′. The expression levels of mRNA were quantified by the way of 2^−ΔΔCq^ and normalized to the internal reference gene GAPDH [25].

#### Statistical analysis

The measured data that collected from ≥3 independent experiments were expressed by mean ± standard deviation and GraphPad Prism 8.0 (GraphPad Software, Inc.) was used to plot the figures. Variations between two groups were verified applying Student’s t-test, and comparisons of differences in more than 2 groups were made by one-way ANOVA followed by Tukey’s post hoc test. Data differences were judged to be statistically significant when p < 0.05.

## Results

We adopted oxygen and glucose deprivation/reoxygenation (OGD/R) to induce R28 cells with the aim of simulating glaucomatous neurodegeneration. Our results show that gastrodin has a protective effect on OGD/ R induced R28 cell injury through activation of PI3K/AKT/Nrf2 signaling pathway, suggesting that gastrodin may have a potential protective effect on retinal I/R injury.

### Gastrodin ameliorated OGD/ R-induced loss of R28 cell viability

CCK-8 assay was used to detect the effects of different concentrations (10 µM, 25 µM, 50 µM and 100 µM) of gastrodin (Figure 1(a)) on R28 cells and the results showed that gastrodin at above concentrations have no obvious effect on the viability of R28 cells (Figure 1(b)). However, OGD/R induction greatly reduced R28 cell viability, indicating that OGD/R model was successfully established. It was noteworthy that gastrodin revived the viability of OGD/R-induced R28 cells in a concentration-dependent manner (Figure 1(c)), and then we detected the effects of gastrodin on the intracellular LDH level of R28 cells with OGD/R induction (Figure 1(d)), and found that there was a marked elevation in intracellular LDH level under OGD/R stimulation (vs Control), inducing significant cytotoxicity, while gastrodin treatment reversed the increase in cytotoxicity induced by OGD/R in a concentration-dependent manner.

**Figure 1.** Gastrodin ameliorated OGD/R-induced the inhibition of R28 cells viability. (a) Chemical formula for Gastrodin. (b) Cell Counting Kit-8 assay detected the effects of different concentrations (10 µM, 25 µM, 50 µM and 100 µM) of gastrodin on R28 cell viability. Effects of gastrodin on OGD/R induced R28 cell viability (c) and LDH level (d). ***P < 0.001 vs. Control; *^##^P* < 0.01 *^###^P* < 0.001 vs OGD/R. OGD/R, oxygen and glucose deprivation/reoxygenation; LDH, lactate dehydrogenase.

### Gastrodin suppressed OGD/R-induced R28 cells apoptosis

To research the impacts of gastrodin on OGD/R-induced apoptosis, R28 cells were cultured in OGD conditions for 4 h and then co-cultured with gastrodin during 24 h reperfusion. Results obtained from TUNEL staining revealed the enhanced OGD/R-induced apoptosis in R28 cells (vs Control); however, gastrodin with different doses dependently reduced the apoptosis of OGD/R-induced R28 cells (Figure 2(a)). Then, under the same treatment conditions, western blot also detected an upregulation of Bax, Cyto-C, c-caspase 9 and c-PARP protein levels as well as a downregulation of Bcl-2 protein level in R28 cells in response to OGD/R stimulation (Figure 2(b)). Interestingly, gastrodin treatment reversed the expressions of these proteins and significantly inhibited the apoptosis induced by OGD/R in R28 cells.

**Figure 2.** Gastrodin suppressed OGD/R-induced R28 cells apoptosis. (a) R28 cell apoptosis was examined adopting TUNEL staining. (b) Expressions of Bcl-2, Bax, Cyto-C, c-caspase 9 and c-PARP proteins were tested via western blot. ***P < 0.001 vs. Control; *^#^P* < 0.05, *^##^P* < 0.01, *^###^P* < 0.001 vs OGD/R. OGD/R, oxygen and glucose deprivation/reoxygenation.

### Gastrodin alleviated OGD/R-induced inflammatory response and oxidative stress of R28 cells

Previous studies have shown that retinal I/R leads to oxidative stress and stimulates excessive production of inflammatory factors and reactive oxygen species, thereby exacerbating neuronal cell death [26,27]. Therefore, we firstly examined the inflammatory cytokines levels and discovered that OGD/R induction remarkably raised the levels of TNF-α, IL-6, and IL-1β as well as their corresponding mRNA levels (vs Control; Figure 3(a-b)). Nevertheless, gastrodin treatment alleviated the expression levels of inflammatory factors TNF-α, IL-6, and IL-1β in OGD/R-induced R28 cells. Subsequently, by further assessing the oxidative stress and antioxidant capacity of the cells, we observed increased malondialdehyde (MDA) level as well as declined activities of glutathione peroxidase (GSH-Px) and superoxide dismutase (SOD) in R28 cells with OGD/R induction (Figure 3(c)). These changes were greatly improved under the treatment of gastrodin. Finally, ROS production in R28 cells was measured (Figure 3(d)). Interestingly, ROS production was increased by OGD/R stimulation (vs Control), while gastrodin with a concentration of 100 µM significantly reduced the ROS production.

**Figure 3.** Gastrodin alleviated OGD/R-induced activation of inflammatory and oxidative stress of R28 cells. RT-qPCR (a) and ELISA (b) kits were used to detect the expression levels of inflammatory factors (TNF-α, IL-6 and IL-1β). (c) Effects of gastrodin on MDA, GSH-Px and SOD levels in OGD/R-induced R28 cells. (d) Fluorescent representative image of ROS in R28 cells. ***P < 0.001 vs. Control; *^#^P* < 0.05, *^##^P* < 0.01, *^###^P* < 0.001 vs OGD/R. OGD/R, oxygen and glucose deprivation/reoxygenation; MDA, malondialdehyde; GSH-Px, glutathione peroxidase; SOD, superoxide dismutase; ROS, reactive oxygen species.

### Gastrodin activated PI3K/AKT/Nrf2 signaling pathway

Activation of PI3K/Akt/Nrf2 signaling pathway could protect retina from oxidative injury induced by ischemia/reperfusion [17,28]. Therefore, we investigated whether PI3K/Akt/Nrf2 signaling pathway is involved in the protective effects of gastrodin on R28 cells. It was clearly observed that OGD/R induction led to apparently inhibited levels of PI3K and AKT phosphorylation. However, 100 µM gastrodin imparted promotive effects on the expressions of p-PI3K and p-AKT in OGD/R-induced R28 cells in comparison with that in OGD/R group, indicating that gastrodin could activate PI3K/AKT/Nrf2 signaling pathway (Figure 4(a-b)).

**Figure 4.** Gastrodin activated the PI3K/AKT/Nrf2 pathway. (a) Western blot was conducted to assay the expressions of PI3K/AKT/Nrf2 signaling pathway. (b) Quantification of PI3K/AKT/Nrf2 signaling pathway related protein expression. **P < 0.01 vs. OGD/R. OGD/R, oxygen and glucose deprivation/reoxygenation.

### PI3K/Akt inhibitor LY294002 reversed the protective effects of gastrodin on OGD/R-induced R28 cell injury

To further verify that gastrodin protected R28 cells from OGD/R-induced damage by activating PI3K/AKT/Nrf2 pathway, OGD/R-R28 cells were co-treated with gastrodin and 10 µM PI3K/Akt inhibitor LY294002. The effects of LY294002 on gastrodin protected R28 cells against OGD/R-induced injury were further observed. It was found that LY294002 administration significantly reduced the protective effects of gastrodin on OGD/R-induced R28 cells (Figure 5(a)), increased intracellular LDH level (Figure 5(b)) and accelerated cell apoptosis (Figure 5(c-d)). Meanwhile, it was also observed that LY294002 reversed the inhibitory effects of gastrodin on OGD/R-induced inflammatory cytokines (TNF-α, IL-6, and IL-1β) (Figure 6(a-b)) and increased MDA level but declined antioxidant GSH-Px and SOD enzyme activities (Figure 6(c)). In addition, in contrast to OGD/R + Gastrodin group, the addition of LY294002 increased the intensity of intracellular ROS green fluorescence and intensified the production of ROS (Figure 6(d)). In conclusion, PI3K/Akt inhibitor LY294002 offset the protective effects of gastrodin on R28 cell viability induced by OGD/R. In other words, gastrodin may play a positive role by activating PI3K/Akt /Nrf2.

**Figure 5.** PI3K/Akt inhibitor reversed the inhibitory effect of Gastrodin on OGD/ R induced apoptosis of R28 cells. Changes in R28 cell viability (a) and LDH level (b) by PI3K/Akt inhibitor. TUNEL staining (c) and western blot (d) were applied for the detection of the effect of PI3K/Akt inhibitor on apoptosis of R28 cells. ***P < 0.001 vs. Control; *^#^P* < 0.05, *^##^P* < 0.01, *^###^P* < 0.001 vs OGD/R. OGD/R, oxygen and glucose deprivation/reoxygenation; LDH, lactate dehydrogenase.

**Figure 6.** PI3K/Akt inhibitor reversed inhibitory effect of Gastrodin on OGD/ R induced inflammation and oxidative stress in R28 cells. (a-b) Changes in TNF-α, IL-6 and IL-1β levels in R28 cells by PI3K/Akt inhibitor. (c) Impacts of PI3K/Akt inhibitor on MDA, GSH-Px and SOD levels in OGD/R-induced R28 cells. (d) ROS fluorescence assay image. ***P < 0.001 vs. Control; *^#^P* < 0.05, *^##^P* < 0.01, *^###^P* < 0.001 vs OGD/R. OGD/R, oxygen and glucose deprivation/reoxygenation; MDA, malondialdehyde; GSH-Px, glutathione peroxidase; SOD, superoxide dismutase; ROS, reactive oxygen species.

## Discussion

Retinal I/R injury is a pathophysiological process of glaucoma [5]. If an effective treatment is not provided, it may cause the loss of retinal function and eventually lead to blindness [29,30]. Neuroinflammation releases a variety of inflammatory factors which play a key role in the pathogenesis of retinal I/R injury, and the induction of oxidative stress and inflammation play a major pathogenic role in the subsequent tissue damage, leading to retinal damage for which there is currently no effective drug treatment [31,32]. It was found that gastrodin extracted from gastrodia elata has a protective effect on retinal ganglion cell injury and that PI3K/AKT/Nrf2 pathway is an important promoter in this action. It was also discovered that gastrodin treatment could significantly improve R28 cell viability, reduce MDA content, improve the activities of SOD and GSH-Px, prevent apoptosis, inhibit the expressions of TNF-α, IL-6, and IL-1β, and reduce ROS level. In terms of mechanism studies, we observed that gastrodin upregulated the expressions of p-Akt, p-P13 K, and Nrf2, while PI3K/Akt inhibitor LY294002 offset the protection of OGD/R-induced R28 cells by gastrodin. This study was the first to discuss the protective function and molecular mechanism of gastrodin in retinal I/R injury model, which offers a new therapeutic avenue for glaucoma research.

Accumulated studies have shown that the anti-inflammatory, antioxidant, and anti-apoptotic pharmacological properties of gastrodin have been proven to have protective effects in myocardial infarction, hypertension, and diabetic retinopathy [12,20,33]. Gastrodin protected retinal ganglion cells in an animal model of acute glaucoma by inhibiting microglia-mediated neuroinflammation [13]. However, its role in retinal I/R injury has not been reported. Therefore, to observe the maximum therapeutic effects of gastrodin on retinal ganglion cell injury, we set up four groups of gastrodin pretreatment with different doses (10 μM, 25 μM, 50 μM, and 100 μM) to evaluate the dose–effect relationship. As expected, gastrodin treatment, even at low doses, significantly improved OGD/R-induced R28 cell damage by inhibiting LDH activity and the releases of pro-inflammatory cytokines, reducing stress-induced changes in MDA, GSH-Px, and SOD, and ultimately inhibiting apoptosis. It is worth considering that gastrodin protected R28 cells from OGD/R-induced damage in a concentration-dependent manner within the concentration range we selected. Therefore, it is necessary to further expand the concentration range of gastrodin to confirm its optimal concentration in the treatment of retinal ganglion cell injury in the following study.

PI3K/AKT/Nrf2 signaling pathway is associated with oxidative stress, inflammation, free radical release, and apoptosis [34–36]. Previous studies have shown that Nrf2 under oxidative stress regulated the expression of stage II detoxification and antioxidant response elements such as glutathione synthase, heme oxygenase-1 (HO-1), and catalase [37], and can be activated through PI3K/Akt pathway to reduce the damage of multiple organs. For example, sulforaphane activated Nrf2 through PI3K/Akt pathway, and improved the liver injury induced by arsenide [38]. Wang et al showed that gastrodin significantly activated the PI3K/Akt pathway and promoted angiogenesis of HUVECs [39]. Xu et al. showed that Edaravone effectively protected the cell viability of H_2_O_2_-treated 661 W cells and improved retinal I/R damage through PI3K/Akt/Nrf2 pathway [18]. Tetrahedral framework nucleic acid prevented retinal I/R injury by activating Akt/Nrf2 pathway [40]. In our study, we found that gastrodin activated PI3K/Akt/Nrf2 pathway as well as reduced oxidative stress and inflammatory factors levels, thereby alleviating OGD/R-induced injury, which was in line with the finding held by Xu et al. [18]. Compared with the results of Wang et al [39]. Our study further expands the application of gastrodin in retinal I/R injury by activating the PI3K/AKT/Nrf2 pathway.

It is noteworthy that there are still some limitations in the present study. First of all, the results of this study are only confirmed by *in vitro* data and further animal experiments were required for *in vivo* verification. Second, we lacked a positive control when evaluating the performance of gastrodin. In addition, the mechanism of gastrodin in retinal I/R injury may not only be related to PI3K/Akt/Nrf2 pathway but other pathways need to be further studied.

## Conclusion

To sum up, gastrodin inhibited retinal ganglion cell damage and reduced intracellular inflammation and oxidative stress levels. In vitro experiments show that gastrodin effectively protected the cell viability of OGD/R-treated R28 cells through PI3K/Akt/Nrf2 pathway. These results suggest that gastrodin has a potential protective effect on retinal I/R injury, which offers a promising direction for clinical treatment of glaucoma.

## Data Availability

The datasets used and/or analyzed during the current study are available from the corresponding author on reasonable request.

## References

[1] Munoz-Negrete FJ, Teus MA, García-Feijoó J, et al. Aniridic glaucoma: an update. Arch Soc Esp Oftalmol (Engl Ed). 2021;96(1):52–59.10.1016/j.oftale.2020.11.01134836589

[2] Torabi R, Harris A, Siesky B, et al. Prevalence rates and risk factors for primary open angle glaucoma in the Middle East. J Ophthalmic Vis Res. 2021;16(4):644–656.3484068710.18502/jovr.v16i4.9755PMC8593541

[3] Zheng Y, Zhang X, Xu X, et al. Deep level set method for optic disc and cup segmentation on fundus images. Biomed Opt Express. 2021;12(11):6969–6983.3485869210.1364/BOE.439713PMC8606159

[4] Conti F, Romano GL, Eandi CM, et al. Brimonidine is neuroprotective in animal paradigm of retinal ganglion cell damage. Front Pharmacol. 2021;12:705405.3436685810.3389/fphar.2021.705405PMC8333612

[5] Yu P, Dong WP, Tang YB, et al. Huperzine A lowers intraocular pressure via the M3 mAChR and provides retinal neuroprotection via the M1 mAChR: a promising agent for the treatment of glaucoma. Ann Transl Med. 2021;9(4):332.3370895910.21037/atm-20-8093PMC7944337

[6] Zhang ZL, Gao Y-G, Zang P, et al. Research progress on mechanism of gastrodin and p-hydroxybenzyl alcohol on central nervous system. Zhongguo Zhong Yao Za Zhi. 2020;45(2):312–320.3223731310.19540/j.cnki.cjcmm.20190730.401

[7] Liu FY, Wen J, Hou J, et al. Gastrodia remodels intestinal microflora to suppress inflammation in mice with early atherosclerosis. Int Immunopharmacol. 2021;96:107758.3416213710.1016/j.intimp.2021.107758

[8] Yuan X, Li Z, Wang X-T, et al. Roles and mechanisms of traditional Chinese medicine and its active ingredients in treating epilepsy. Zhongguo Zhong Yao Za Zhi. 2019;44(1):9–18.3086880610.19540/j.cnki.cjcmm.20181012.006

[9] Sun W, Lu H, Lyu L, et al. Gastrodin ameliorates microvascular reperfusion injury-induced pyroptosis by regulating the NLRP3/caspase-1 pathway. J Physiol Biochem. 2019;75(4):531–547.3144098710.1007/s13105-019-00702-7

[10] Peng Z, Wang S, Chen G, et al. Gastrodin alleviates cerebral ischemic damage in mice by improving anti-oxidant and anti-inflammation activities and inhibiting apoptosis pathway. Neurochem Res. 2015;40(4):661–673.2558291610.1007/s11064-015-1513-5

[11] Li S, Bian L, Fu X, et al. Gastrodin pretreatment alleviates rat brain injury caused by cerebral ischemic-reperfusion. Brain Res. 2019;1712:207–216.3074280810.1016/j.brainres.2019.02.006

[12] Zhang TH, Huang C-M, Gao X, et al. Gastrodin inhibits high glucose induced human retinal endothelial cell apoptosis by regulating the SIRT1/TLR4/NFkappaBp65 signaling pathway. Mol Med Rep. 2018;17(6):7774–7780.2962026710.3892/mmr.2018.8841

[13] Wang JW, Liu Y-M, Zhao X-F, et al. Gastrodin protects retinal ganglion cells through inhibiting microglial-mediated neuroinflammation in an acute ocular hypertension model. Int J Ophthalmol. 2017;10(10):1483–1489.2906276410.18240/ijo.2017.10.01PMC5638966

[14] Hu Q, Zhang W, Wu Z, et al. Baicalin and the liver-gut system: pharmacological bases explaining its therapeutic effects. Pharmacol Res. 2021;165:105444.3349365710.1016/j.phrs.2021.105444

[15] Sun X, Chen L, He Z. PI3K/Akt-Nrf2 and anti-inflammation effect of macrolides in chronic obstructive pulmonary disease. Curr Drug Metab. 2019;20(4):301–304.3082723310.2174/1389200220666190227224748

[16] Wu Y, Qiu G, Zhang H, et al. Dexmedetomidine alleviates hepatic ischaemia-reperfusion injury via the PI3K/AKT/Nrf2-NLRP3 pathway. J Cell Mol Med. 2021;25(21):9983–9994.3466441210.1111/jcmm.16871PMC8572787

[17] Chen S, Li X, Wang Y, et al. Ginsenoside Rb1 attenuates intestinal ischemia/reperfusion induced inflammation and oxidative stress via activation of the PI3K/Akt/Nrf2 signaling pathway. Mol Med Rep. 2019;19(5):3633–3641.3086472510.3892/mmr.2019.10018PMC6471656

[18] Xu YP, Han F, Tan J. Edaravone protects the retina against ischemia/reperfusion induced oxidative injury through the PI3K/Akt/Nrf2 pathway. Mol Med Rep. 2017;16(6):9210–9216.2903949710.3892/mmr.2017.7739

[19] Li X, Zhu Q, Liu Y, et al. Gastrodin protects myocardial cells against hypoxia/reoxygenation injury in neonatal rats by inhibiting cell autophagy through the activation of mTOR signals in PI3K-Akt pathway. J Pharm Pharmacol. 2018;70(2):259–267.2914806810.1111/jphp.12838

[20] Xing Y, Li L. Gastrodin protects rat cardiomyocytes H9c2 from hypoxia-induced injury by up-regulation of microRNA-21. Int J Biochem Cell Biol. 2019;109:8–16.3068456910.1016/j.biocel.2019.01.013

[21] Yuan B, Huang H, Qu S, et al. Gastrodin pretreatment protects liver against ischemia-reperfusion injury via activation of the Nrf2/HO-1 pathway. Am J Chin Med. 2020;48(5):1159–1178.3266897310.1142/S0192415X20500573

[22] Sun Q, Zhang T, Xiao Q, et al. Procyanidin B2 inhibits angiogenesis and cell growth in oral squamous cell carcinoma cells through the vascular endothelial growth factor (VEGF)/VEGF receptor 2 (VEGFR2) pathway. Bioengineered. 2022;13(3):6500–6508.3522089610.1080/21655979.2022.2033013PMC8973926

[23] Zeng K, Xi W, Qiao Y, et al. Paeoniflorin inhibits epithelial mesenchymal transformation and oxidative damage of lens epithelial cells in diabetic cataract via sirtuin 1 upregulation. Bioengineered. 2022;13(3):5903–5914.3518465310.1080/21655979.2021.2018534PMC8974002

[24] Ding L, and Li J. FXYD domain containing ion transport regulator 5 (FXYD5) silencing promotes cell viability and alleviates inflammatory response in cerulein-induced AR42J cells by blocking JAK2/STAT3 signaling pathway. Bioengineered. 2022;13(2):2639–2647.3504243610.1080/21655979.2021.2023795PMC8974200

[25] Hirschfeld M, Ge I, Rücker G, et al. Mutually distinguishing microRNA signatures of breast, ovarian and endometrial cancers in vitro. Mol Med Rep. 2020;22(5):4048–4060.3300025910.3892/mmr.2020.11466

[26] Ryu J, Gulamhusein H, Oh JK, et al. Nutrigenetic reprogramming of oxidative stress. Taiwan J Ophthalmol. 2021;11(3):207–215.3470373510.4103/tjo.tjo_4_21PMC8493979

[27] Scheid S, Goeller M, Baar W, et al. Hydrogen sulfide reduces ischemia and reperfusion injury in neuronal cells in a dose- and time-dependent manner. Int J Mol Sci. 2021;22(18):10099.3457625910.3390/ijms221810099PMC8467989

[28] Hu S, Wu Y, Zhao B, et al. Panax notoginseng saponins protect cerebral microvascular endothelial cells against oxygen-glucose deprivation/reperfusion-induced barrier dysfunction via activation of PI3K/Akt/Nrf2 antioxidant signaling pathway. Molecules. 2018;23(11):2781.10.3390/molecules23112781PMC627853030373188

[29] Guan L, Li C, Zhang Y, et al. Puerarin ameliorates retinal ganglion cell damage induced by retinal ischemia/reperfusion through inhibiting the activation of TLR4/NLRP3 inflammasome. Life Sci. 2020;256:117935.3252628610.1016/j.lfs.2020.117935

[30] Zadeh JK, Garcia-Bardon A, Hartmann EK, et al. Short-time ocular ischemia induces vascular endothelial dysfunction and ganglion cell loss in the pig retina. Int J Mol Sci. 2019;20(19):4685.10.3390/ijms20194685PMC680151531546635

[31] Deng C, Chen S, Li X, et al. Role of the PGE2 receptor in ischemia-reperfusion injury of the rat retina. Mol Vis. 2020;26:36–47.32165825PMC7043643

[32] Zhou X, Lv J, Li G, et al. Rescue the retina after the ischemic injury by polymer-mediated intracellular superoxide dismutase delivery. Biomaterials. 2021;268:120600.3336050710.1016/j.biomaterials.2020.120600

[33] Qian L, Yan S, Li Y, et al. The effects of gastrodin injection on hypertension: a systematic review and meta-analysis. Medicine (Baltimore). 2020;99(27):e20936.3262969510.1097/MD.0000000000020936PMC7337477

[34] Xiong J Yang J, Yan K, et al. Ginsenoside Rk1 protects human melanocytes from H2O2induced oxidative injury via regulation of the PI3K/AKT/Nrf2/HO1 pathway. Mol Med Rep. 2021;24(5). DOI:10.3892/mmr.2021.12462.PMC848512034558653

[35] Kohandel Z, Farkhondeh T, Aschner M, et al. Anti-inflammatory action of astaxanthin and its use in the treatment of various diseases. Biomed Pharmacother. 2021;145:112179.3473607610.1016/j.biopha.2021.112179

[36] Fu Z, Jiang Z, Guo G, et al. rhKGF-2 attenuates smoke inhalation lung injury of rats via activating PI3K/Akt/Nrf2 and repressing FoxO1-NLRP3 inflammasome. Front Pharmacol. 2021;12:641308.3436683810.3389/fphar.2021.641308PMC8339412

[37] Alvarez-Lerma F, Palomar M, Villasboa A, et al. Epidemiological study of clostridium difficile infection in critical patients admitted to the intensive care unit. Med Intensiva. 2014;38(9):558–566.2450333110.1016/j.medin.2013.11.007

[38] Thangapandiyan S, Ramesh M, Hema T, et al. Sulforaphane potentially ameliorates arsenic induced hepatotoxicity in albino wistar rats: implication of PI3K/Akt/Nrf2 signaling pathway. Cell Physiol Biochem. 2019;52(5):1203–1222.3100196010.33594/000000082

[39] Wang J, Wu M . The up-regulation of miR-21 by gastrodin to promote the angiogenesis ability of human umbilical vein endothelial cells by activating the signaling pathway of PI3K/Akt. Bioengineered. 2021;12(1):5402–5410.3442481310.1080/21655979.2021.1964895PMC8806924

[40] Qin X, Li N, Zhang M, et al. Tetrahedral framework nucleic acids prevent retina ischemia-reperfusion injury from oxidative stress via activating the Akt/Nrf2 pathway. Nanoscale. 2019;11(43):20667–20675.3164245210.1039/c9nr07171g

